# Keratoconus Severity Classification Using Features Selection and Machine Learning Algorithms

**DOI:** 10.1155/2021/9979560

**Published:** 2021-11-16

**Authors:** Mustapha Aatila, Mohamed Lachgar, Hrimech Hamid, Ali Kartit

**Affiliations:** ^1^LTI Laboratory, ENSA, Chouaib Doukkali University, El Jadida 1166, Morocco; ^2^Analysis and Modeling of Systems and Decision Support Laboratory, ENSA of Berrechid, Hassan 1er University of Settat, Berrechid 218, Morocco

## Abstract

Keratoconus is a noninflammatory disease characterized by thinning and bulging of the cornea, generally appearing during adolescence and slowly progressing, causing vision impairment. However, the detection of keratoconus remains difficult in the early stages of the disease because the patient does not feel any pain. Therefore, the development of a method for detecting this disease based on machine and deep learning methods is necessary for early detection in order to provide the appropriate treatment as early as possible to patients. Thus, the objective of this work is to determine the most relevant parameters with respect to the different classifiers used for keratoconus classification based on the keratoconus dataset of Harvard Dataverse. A total of 446 parameters are analyzed out of 3162 observations by 11 different feature selection algorithms. Obtained results showed that sequential forward selection (SFS) method provided a subset of 10 most relevant variables, thus, generating the highest classification performance by the application of random forest (RF) classifier, with an accuracy of 98% and 95% considering 2 and 4 keratoconus classes, respectively. Found classification accuracy applying RF classifier on the selected variables using SFS method achieves the accuracy obtained using all features of the original dataset.

## 1. Introduction

In many fields (computer vision, pattern recognition,…, etc.), the resolution of most problems is based on the processing of data extracted from data acquired in the real world and structured in the form of vectors [1]. The quality of the processing system depends directly on the right choice of the content of these vectors. But, in many cases, the resolution of the problem becomes almost impossible because of the very large dimension of these vectors. Therefore, it is often useful, and sometimes necessary, to proceed to a selection of the most relevant features compared to the used resolution method, by eliminating harmful features to the adopted system, even if this selection of variables may lead to a slight loss of information. Moreover, to extract important features from these large variables and data, statistical techniques were used to minimize noise and redundant data [2]. Thus, the selection of parameters is really important in improving the model and this is by using correlated and nonredundant parameters. In addition, learning is done quickly, and the complexity of the model will be reduced, making it easier to understand and improving metric performance in terms of precision, accuracy, and recall [3].

There are four important reasons why feature selection is essential. First, spare the model to reduce the number of parameters. Second, to decrease the learning time. Then, to reduce overfilling by improving the generalization and to avoid the problems of dimensionality [4]. So, our motivation is to get the best model with high predictions and small errors.

It is in this context particularly that this work is presented that consists in determining the most relevant parameters for diagnosing keratoconus, which corresponds to a deformation of the cornea (the transparent coating of the iris and the pupil of the eye) which gradually thins [5], loses its normal spherical shape, and takes on an irregular cone shape as illustrated in Figure 1 below.

Keratoconus can be diagnosed during a consultation, motivated by the existence of functional signs secondary to progressive irregular myopic astigmatism. In general, the functional signs are not very specific. The most common is the presence of visual blurring, photophobia, fog, progressive loss of visual acuity predominantly at a distance, monocular diplopia, or persistent irritation [7]. However, there are several tools to diagnose keratoconus such as corneal topography, corneal biomechanics, and optical coherence tomography OCT. Each tool has its own parameters to diagnose the disease, so in this study, we will analyze the different parameters using machine learning algorithms, then, a validation of obtained results by a physician expert in the field will be performed. In this work, feature selection techniques are used to increase the potential for classifier generalization. Thus, a comparison of the results without and with feature selection, using filters, wrappers, embedded, and hybrid methods, will also be presented. The main contributions of this research are summarized as follows. First, the analysis of various parameters extracts the most relevant ones, especially for the analysis of classification data. Second, a comparative study of different machine learning models, such as random forest (RF), support vector machine (SVM), *K*-nearest neighbors (KNN), decision tree (DT), Naive Bayes (NB), logistic regression (LR), and linear discriminant analysis (LDA) using critical features. Different models will have different strengths in classifying data which will affect classification performance. Also, multiple feature selection methods are used to get the best accuracy. In addition, we mainly review the variable selection application and provide description, analysis, and future research suggestions. The remain of this paper is organized as follows. The following section represents the related works.  Section 3 describes the employed methodology in keratoconus classification. The simulation results are presented in Section 4.  Section 5 presents the result discussion. Finally, the conclusions and future directions of the research are indicated in Section 6.

## 2. Related Works

Artificial intelligence (AI) has integrated different domains of medicine field such as ophthalmology. The number of works that focused on the detection of ophthalmic diseases using machine learning (ML) is growing. Several research teams aim to build intelligent systems for keratoconus diagnosis and classification. In [8], authors proposed an ensemble of deep transfer learning considering SqueezeNet (SqN), AlexNet (AlN), ShuffleNet (SfN), and MobileNet-v2 (MbN) for improved detection of keratoconus. Built system was trained on a dataset of 2136 corneal topographic maps and provided an accuracy in the range of 92.2% to 94.8%. To evaluate keratoconus diagnosability, the authors of [9] developed an intelligent system based on deep learning using color-coded map with Placido disk-based corneal topography. Trained on a total of 3390 color-coded map images representing 4 eyes classes, the proposed system achieved an accuracy of 78.5% in keratoconus classification. Authors of [10] proposed an intelligent system based on time delay neural network (TDNN) to verify both the progression predictability using two prior tomography measurements and the system accuracy when labelling the eye as stable or suspect progressive. Obtained results showed a sensitivity of 70.8% and a specificity of 80.6% using data of 743 patients captured by Pentacam. To screen keratoconus using corneal topography, authors of [11] adopted three convolutional neural network (CNN) models (VGG16, InceptionV3, and ResNet152) to develop the proposed system. Trained on a dataset of 354 images, built system achieved accuracies 93.1%, 93.1%, and 95.8% using VGG16, InceptionV3, and ResNet152, respectively. The authors of [12] proposed a convolutional neural network- (CNN-) based intelligent system for keratoconus detection. Trained on a data set of 3000 images, provided by Pentacam technology only, developed system provided a classification with an accuracy of 99.33%. Authors of [13] built feedforward neural network- (FNN-) based intelligent system for keratoconus identification. Developed system discriminate keratoconus eyes with an accuracy of 96.56% on a dataset of 851 elements using neighborhood component analysis for features selection (NCAFS). In [14], a RF model was used to detect keratoconus. The obtained system provided a classification accuracy of 76% on a dataset of 500 images. Using a dataset of 124 images and using 29 parameters, the authors of [15] have developed a keratoconus identification and classification system using Bayesian neural networks (BNN). Adopting principal component analysis (PCA) of features selection, the developed system allowed a classification with an accuracy of 73% and 80%, respectively, for supervised and unsupervised learning. In [5], the authors proposed a keratoconus classification system based on unsupervised machine learning (UnML) and trained on a dataset of 3156 images. To reduce the dimensionality of the input data from 420 to eight important variables, the authors adopted the PCA method. The built system allowed keratoconus identification with a specificity of 94.1% and a sensitivity of 97.7%. In [16], authors have developed a BNN-based system of keratoconus classification. Classification accuracy of this system, using 16 parameters on a dataset of 60 elements, was 100%. The authors of [17] have built an intelligent system to classify keratoconus based on CNN technique. Trained on a dataset of 543 images, the accuracy of the proposed system was 99.1%. In [18], the authors developed SVM-based system for keratoconus detection and classification. Classification accuracy of built system was between 92.6% and 98.0% on a dataset of 131 images and 25 extracted parameters. Trained on a dataset of 372 images using 55 parameters, the system proposed in [19] allowed keratoconus classification using decision trees (DT) model. Developed system discriminated normal and keratoconus eyes with a sensitivity of 100% and a specificity of 99.5% and classified normal and forme fruste keratoconus eyes with 93.6% sensitivity and 97.2% specificity. The authors of [20] proposed an SVM-based system for keratoconus detection and classification. Classification accuracy provided by the built system was 98.2% on a dataset of 3502 elements and using 7 parameters. In [21], authors have developed a classification system for keratoconus with an accuracy of 90% on a dataset of 40 images and 12 parameters. The authors of [22] have proposed eight classifiers in order to compare their performance. Using 11 extracted parameters on a dataset of 88 elements, RF, SVM, KNN, logistic regression (LR), linear discriminant analysis (LDA), lasso regression (LaR), DT, and multilayer perceptron neural network (MPAN) models provided an accuracy of 87%, 86%, 73%, 81%, 81%, 84%, 80%, and 52%, respectively. The authors of [23] developed a system for early and mild keratoconus detection. Based on logistic regression, this system allowed early and mild keratoconus detection using only 5 selected variables from a dataset of 27 features. The variable selection was performed using *χ*^2^ and Kruskal-Wallis algorithms. The overall accuracy of this system was 73%. In [24], the authors have proposed a comparative study of 25 different machine learning models allowing keratoconus detection based on the corneal imaging. Different classifiers were trained on a dataset of 3151 corneal images, collected from 3146 eyes. Applied on a subset of 8 selected parameters using subset selection (SS) and feature ranking (FRank) feature selection methods, proposed models provided classification accuracy varying between 62% and 94%, and the highest performance was generated by the SVM model.  Table 1 below summarizes the works already cited:

Despite the good performance of different systems already mentioned in the related works, which allowed a very good discrimination between normal and keratoconus eyes in keratoconus classification, many works of them did not mention that they used variable selection method. Such methods could increase system performance, by eliminating irrelevant variables, reducing data dimensionality, and optimizing algorithm prediction time. In this work, we propose a comparative study of keratoconus classification using different classifiers, without and with features selection, by applying different types of variables selection algorithms.

## 3. Methodology

### 3.1. Feature Selection

The performance of a machine learning system is affected by several factors, including the representation and relevance of the data used by that system. Generally, not all learning data is always relevant to the system. However, the selection of relevant features, by eliminating less informative, redundant, or even irrelevant variables, is of great importance to the learning system. The feature selection model adopted in this work is described in Figure 2 below.

### 3.2. Data Preprocessing

The data preprocessing stage consists generally of eliminating irrelevant and redundant variables, handling missing values in the dataset, and handling categorical data, such as textual data that is difficult to understand for machines. The dataset resulting from this step is then used by different types of algorithms in order to select relevant features.

### 3.3. Filters

First, the used dataset was filtered using the filters. These methods allow to select variables using different approaches and criteria to calculate the relevance of a variable before the learning phase. In other words, the evaluation of the importance of characteristics is done independently of the use of a classifier. However, the characteristics retained by the filters can be used by all learning algorithms. Filters remove irrelevant, redundant, constant, duplicated, and correlated characteristics in a very efficient manner [25]. The main filtering methods used in this work are:

1. Fast correlation-based filter (FCBF) that allows to select features representing a low correlation with other features and which are more correlated to the target variable using symmetrical uncertainty [26]
2. Mutual information (MI) which can be defined as the measure of reduction of uncertainty of a variable in view of the knowledge of a second variable. It represents a statistical dependence between two random variables, thus, measuring their degree of dependence in the probabilistic sense [25]
3. Analysis of variance (ANOVA) is a statistical model that allows to compare the mathematical expectation of several subsamples in order to demonstrate the possible similarities or differences on specific aspects in a studied sample [27]
4. Variance algorithm calculates the variance of different features. This algorithm selects the features for which the variance is greater or equal to a special threshold *t* defined initially

### 3.4. Wrapper Methods

The weakness of filters is the fact that they do not consider the learning algorithm when selecting variables. Wrapper methods solve this problem by introducing the learning algorithm during feature selection. This method evaluates the classification performance of a subset of variables during the selection procedure using a classifier [25]. The wrapper algorithms used in this study are:

1. Recursive feature elimination (RFE) is a selection feature algorithm in which specific weight values are assigned to features by application of external estimator. This process is repeated recursively, and in each step, attributes whose weights are the smallest ones are removed from the current set. It works until the desired set of features to select from is eventually reached. In the RFE approach, the number of features to select should be initially defined [28]
2. Sequential forward selection (SFS) is an iterative algorithm starting from an empty subset of variables. For each iteration, FFS algorithm evaluates the variables individually and retains the variable that best improves the model. The selection process stops when the performance of the system is no longer increased by adding a new variable [29]
3. Sequential backward selection (SBS) is an iterative algorithm initially using all the features of the dataset. BFE eliminates the least significant variable in each iteration until no performance improvement is noticed [29]
4. Genetic algorithms (GA) are iterative algorithms based on the genetic evolution process. GA constitutes chromosomes from an initial population by proposing potential solutions to the studied problem. This initial population of solution evolves using three operators (selection, crossing, and mutation operators) to converge to the best solution [30]
5. Hybrid recursive feature addition (HRFA) creates a model using only the most relevant variable selected by ranking different variables of the original dataset. The algorithm adds the most important feature at each step and reassesses the performance of the model [31]. If the metric exceeds an arbitrarily defined threshold, the variable is retained otherwise it can be deleted. This processing is repeated until all variables are evaluated

The feature subset selected by a wrapper method represents a strong dependence on the classifier used in the selection phase. However, changing the classification algorithm can produce poor classification performance.

### 3.5. Embedded Methods

Embedded methods select the features judged critical during the training of the machine learning model adopted for the classification [32].

### 3.6. Hybrid Method

Hybrid method is a combination of a filter and a wrapper method of features selection. The features retained using the filter algorithm are evaluated by the wrapper algorithm to find the best subset of features [25].

Choosing the right method for selecting features usually depends on the initial goal. Filters are very good in reducing data size and eliminating redundant features. Wrapper methods on the other hand are very powerful at producing good classification precision using a given classifier.  Table 2 below illustrates different types of feature selection algorithms used in this study:

### 3.7. Classification Methodology

The main objective of this work is to compare performance and execution time of different machine learning models in the classification of keratoconus. Classification is realized in first time using all features of the dataset of keratoconus, available in Harvard Dataverse [33]. In the second time, the classification is performed after a selection of crucial features by the application of different types of feature selection algorithms already cited on the original dataset. In other words, keratoconus classification is realized using different models with and without feature selection. The 10-fold cross-validation technique has been commonly used for different machine learning models in order to avoid the overfitting problem.  Figure 3 below illustrates the classification methodology adopted in this study.

Random forest (RF) is an ensemble of many individual decision trees. It is a classification prediction method which is based on decision trees. This method is proposed by Breiman in 2001 [34]. RF is one of ensemble methods that involve using many learners to improve the performance of any single one of them individually. This method can be described as technique that uses a combination of a group of weak decision trees together, to create a stronger and aggregated one. The classification algorithm of RF is structured as follows [35].

If the data change a little, the performances the individual trees may change but the forest is relatively stable because it is a combination of many trees, and this is the main advantage of RF.

Naive Bayes (NB) technique is based on the Bayes theorem. The Naïve Bayes is a probabilistic classifier which is well suited for high dimensional datasets. Despite of its simplicity, NB algorithm can outstrip more efficient other classifiers. NB classifier computes probability estimates rather than predictions. To verify whether a given observation belongs to a specific class, NB algorithm calculates probability each output value. NB assumes that the attributes present do not influence each other and are mutually independent [36]. This is called conditional independence.

Consider a dataset *D* composed of *N* attributes, and each tuple of *D* is structured in *N* values. Suppose that *C*1 and *C*2 are the two available class labels for the target data. For each new tuple *X*, NB classifier predict that *X* ∈ Ci if the class Ci has a highest probability condition on *X*, i.e.,

(1) $$\begin{array}{c} \text{If }P\left(\frac{C_{i}}{X}\right)>P\left(\frac{C_{j}}{X}\right)\text{where }1\leq j\leq m. \end{array}$$

If the class Ci had the maximum probability which *P*(Ci/*x*) is maximized, this class is called maximum posterior hypothesis. As *P*(*X*) is constant for all the classes the equation can be depicted as:

(2) $$\begin{array}{c} P\left(\frac{C_{i}}{x}\right)=P\left(\frac{X}{C_{i}}\right)*P\left(C_{i}\right). \end{array}$$

*K*-nearest neighbor (KNN) algorithm is a simple and easy supervised machine learning algorithm that can be used to solve classification and regression problems. According to the measure of similarity, like the distance functions, *K*-NN provides a classification of the new cases, by attributing them to the most present category among these *K* neighbors [37].

The distance of the case to be classified to the other cases is ensured using some norm-based measurement functions, such as

(3) $$\begin{array}{c} \text{Euclidean distances}:\sqrt{\overset{n}{\underset{i=1}{\sum }}{\left(x_{i}-y_{i}\right)}^{2}}, \end{array}$$

(4) $$\begin{array}{c} \text{or Manhattan distances}:\overset{n}{\underset{i=1}{\sum }}\left|x_{i}-y_{i}\right|. \end{array}$$

The *K*-NN algorithm can be described as follows [38].

Logistic regression (LR) is a statistical-based classification model, and it is a linear predictive algorithm based on the concept of probability. The decision rule of the LR is ensured by a complex function called Sigmoid function. The probability generated by Sigmoid function is limited between 0 and 1. When the predicted value is greater than a threshold, the event is likely to occur, while when this value is below the same threshold, it is not [39]. The Sigmoid function is defined as follows:

(5) $$\begin{array}{c} P\left(\left.Y\right|X\right)=\frac{1}{1+e^{-f\left(x\right)}}, \end{array}$$

(6) $$\begin{array}{c} f\left(x\right)=x_{0}+x_{1}\beta_{1}+\cdots +x_{k}\beta_{k}+\varepsilon , \end{array}$$

where *x*_*j*_ and *β*_*j*_ are the features and their corresponding weights/coefficients.

Linear discriminant analysis (LDA) is a supervised classification technique belonging to competitive machine learning models, developed in 1936 by R. A. Fisher. It is a simple and robust classification method which produces models that provide a good accuracy as more complex methods [40]. The idea behind LDA is to search a linear combination of variables (predictors) that best separates two classes (targets). Linear discriminant analysis process can be described into 5 steps as follows [40].

The within-class scatter matrix is calculated using the following mathematical equation [40]:

(7) $$\begin{array}{c} S_{W}=\overset{c}{\underset{i=1}{\sum }}S_{i}, \end{array}$$

where *c* is the total number of distinct classes and

(8) $$\begin{array}{c} S_{i}=\overset{n}{\underset{x\in D_{i}}{\sum }}\left(x-m_{i}\right){\left(x-m_{i}\right)}^{T}, \end{array}$$

and

(9) $$\begin{array}{c} m_{i}=\frac{1}{n_{i}}\overset{n}{\underset{x\in D_{i}}{\sum }}x_{k}, \end{array}$$

where *x* is a sample (a row) and *n* is the total number of samples within a given class.

The between-class scatter matrix is calculated using the following mathematical equation:

(10) $$\begin{array}{c} S_{B}=\overset{c}{\underset{i=1}{\sum }}N_{i}\left(m_{i}-m\right){\left(m_{i}-m\right)}^{T}, \end{array}$$

where

(11) $$\begin{array}{c} m_{i}=\frac{1}{n_{i}}\overset{n}{\underset{x\in D_{i}}{\sum }}x_{k}, \end{array}$$

(12) $$\begin{array}{c} m=\frac{1}{n}\overset{n}{\underset{i}{\sum }}x_{i}. \end{array}$$

The linear discriminants are provided by solving the generalized eigenvalue problem of the following matrix:

(13) $$\begin{array}{c} S_{W}^{-1}S_{B}. \end{array}$$

Decision tree (DT) is a tree-structured classification model. Each node of a DT represents a test evaluating an attribute of any individual in the population. The arcs from a node represent the responses to the test associated with this node. Each sheet of DT corresponds to a class, called the default class. The DT used in this work is based on the CART algorithm presented below [41].

Support vector machine (SVM) consists in finding a hyperplane (straight line in the case of two dimensions) that best separates these two classes in the case of a binary classification [42]. The separating hyperplane is represented by the following equation [43]:

(14) $$\begin{array}{c} H\left(x\right)=w^{T}x+b, \end{array}$$

where *w* is a vector of *m* dimensions and *b* is a term. The decision function, for an example *x*, can be expressed as follows:

(15) $$\begin{array}{c} \left\{\begin{array}{cc} \text{Class}=1 & Si\;H\left(x\right)>0,\\ \text{Class}=-1 & Si\;H\left(x\right)<0. \end{array}\right. \end{array}$$

In reality, most of the problems are multiclass; in this case, solutions based on SVM methods reduce the multiclass problem to a composition of several biclass hyperplanes making it possible to draw the decision boundaries between the different classes.

### 3.8. Evaluation Metrics

In different steps of keratoconus classification, the performance evaluation of obtained results is based in classification accuracy, recall, *f*1-score, ROC curve, and prediction time.

The precision is a measure that expresses how accurate your model is relatively to those predicted positive, how many of them are actually positive [44]. In our case, precision indicates eyes correctly predicted having keratoconus out of all eyes actually having keratoconus. Precision is calculated using the following formula:

(16) $$\begin{array}{c} \text{Precision}=\frac{\text{TP}}{\text{TP}+\text{FP}}. \end{array}$$

The recall (or true positive rate) is the measure of our model correctly identifying true positives [44]. Thus, for all instances who actually have keratoconus disease, recall tells indicates how many the model correctly identified as having a keratoconus disease. Recall is computed using the following equation:

(17) $$\begin{array}{c} \text{Recall}=\frac{\text{ TP}}{\text{TP}+\text{FN}}. \end{array}$$

The *f*1-score is a metric combining false positives and false negatives to strike a balance between precision and recall [44]. It is a weighted average (or harmonic average) of the precision and recall. Model is considered perfect when *F*1-score is 1, while the model is considered as a total failure when *F*1-score is 0. *F*1-score is computed as follows:

(18) $$\begin{array}{c} F1-\text{Score}=2*\frac{\text{ Precision}*\text{Recall }}{\text{ Precision}+\text{Recall }}. \end{array}$$

The accuracy is a popular measure that describes classification performance of the model over all classes [44]. It represents the ratio between the number of correct predictions to the total number of predictions. Accuracy is calculated using the following equation:

(19) $$\begin{array}{c} \text{Accuracy}=\frac{\text{TP}+\text{TN}}{\text{TP}+\text{TN}+\text{FP}+\text{FN}}, \end{array}$$

where true positives (TP) is number of correct samples predicted as “yes.” True negatives (TN) is number of correct samples predicted as “no.” False positives (FP) is number of samples that are incorrectly predicted as “yes” when they are actually “no.” False negatives (FN) is number of samples that are incorrectly predicted as “no” when they are actually “yes.”

Execution time is the measurement of the time consumed by different machine learning models for the training and prediction phases to perform a classification.

Area under ROC curve (AUC) curve is a graph that represents relationship between false positive rate and true positive rate of a test for all possible thresholds. Ordinates represent false positive rate and abscissas correspond to true positive rate. ROC curve expresses the ability of a classifier to differentiate between true positive (TP) and false positive (FP) rates [44]. The value of ROC lies between 0.5 and 1, and efficient classifier tends to maximize the ROC value towards 1.

## 4. Simulation Results

### 4.1. Dataset Description

The current comparative study is based on the public keratoconus dataset of Harvard Dataverse [33], available in: https://dataverse.harvard.edu/dataset.xhtml?persistentId=doi:10.7910/DVN/G2CRMO. Structured in csv file, this dataset is composed of 446 features of 3162 rows. Eyes are classified in 4 classes as described in Table 3 below.

This dataset is extracted and used in [5] from a dataset of 12,242 eye images acquired from SS-1000 CASIA OCT Imaging Systems images and representing corneal swept source optical coherence tomography (OCT) in multiple centers across Japan.

### 4.2. Technical Description of the Used Calculator

The different classification models studied were implemented in Python using Jupyter application. All the simulations were carried out with CUDA 10.1 under Ubunto16.04, using a Xeon E5-2697 V4 CPU (18 cores, 36 threads) ECC: on, a RAM of 64 Gbytes DDR4 2133 MHz, a GPU 1 GTX 1070 Ti (8GB GDDR5, CUDA cores: 2432), total 38912 threads, ECC: off and a 2 Tesla k80 GPU (24 GB GDDR5, CUDA cores: 4992), total 53,248 threads, ECC: on.

### 4.3. Obtained Results considering Two Classes

Obtained results of first classification task, applying different algorithms of features selection on the original dataset, considering just two classes of eyes (class 1 for normal eyes with a total of 264 elements, and class 2 of keratoconus eyes with à total of 2989 elements) and using different classification models are illustrated in Figures 4–6 below.

Figures 7–9 show the classifier performance comparison based on the accuracy, using retained features by different features selection methods and considering 2 keratoconus classes.

### 4.4. Obtained Results considering Four Keratoconus Classes

The same proposed model is evaluated using the original dataset and considering the four classes of eyes as already illustrated in Table 2, both without and with features selection. Figures 10 and 11 below represent simulation results.

The classification algorithm comparison based on the classification accuracy of different models associated to the classification task considering 4 keratoconus classes is illustrated in Figures 12 and 13 below.

The results provided by the previous simulations show that the random forest algorithm represents the highest performance compared to other algorithms, both with and without features selection. RF algorithm allowed keratoconus classification with an accuracy around 98% in the case of classification according to 2 classes and exceeding 91% in the case of the classification considering 4 keratoconus classes. These results are obtained by using a number of variables to be retained fixed at a maximum of 10 for the features selection algorithms which require mentioning the number of features to be selected.

## 5. Discussion

The main objective of this work is to present a comparative study of different machine learning models' performances in the case of keratoconus classification, based on the public keratoconus dataset of Harvard Dataverse, both without and with feature selection. Each classification technique was applied using all the variables of the dataset, then by applying 11 features selection algorithms to select relevant variables. To assess studied model's ability to correctly classify keratoconus, 2 classification tasks were performed. The first classification was carried out retaining only 2 classes (normal eyes and keratoconus eyes), and the second classification was carried out considering 4 classes (class 1 for normal eyes, class 2 for healthy eyes with form fruste keratoconus, class 3 for eyes with mild keratoconus, and class 4 for eyes with advanced keratoconus stage).

In overall, RF algorithm has a good ability of differentiating between normal eyes and keratoconus eyes. RF classifier provided the best performance in terms of classification accuracy using all features and for all algorithms of variable selection accepted the filter combined to the HRFA algorithm in the case of 2 and 4 classes of keratoconus.  Table 4 below shows the performance of RF model in terms of classification accuracy retaining 2 and 4 keratoconus classes with respect to the different algorithms of features selection already mentioned.

On the other hand, and as illustrated by Table 2 below, RF algorithm represented the highest performances by the application of the SFS algorithm of feature selection. In the case of the classification using only 2 eye classes, this method generated an accuracy of 98.10% using just 10 variables, against 98.0% by the same classifier applied to all the dataset composed of 446 variables. Also, the execution time in this case was reduced remarkably from 16.014 seconds to 3.241 seconds. In the second classification task, taking into account 4 classes of keratoconus, the classification accuracy of the RF was of the order of 95.32% by processing the 10 selected variables using the SFS algorithm, against 95.32% by use of all dataset variables with a significant decrease in execution time from 20.485 seconds to 3.702 seconds.

Table 5 below illustrates the performances of different classifiers, applied with different techniques of features selection, considering 2 and 4 classes.

Generally, algorithms of RF, LR, and LDA represent the best performances in different keratoconus classification tasks.  Figure 14 below illustrates the ROC curves comparison of RF, LR, and LDA algorithms applied on the retained variables, using SFS features selection algorithm, with respect to the keratoconus classes C1, C2, C3, and C4.

Obtained ROC curves show that RF, LR, and LDA models discriminate accurately different classes of keratoconus using just 10 variables instead of 446 features, hence, the effectiveness of SFS algorithm in the selection of relevant variables, thus, reducing the execution time and material resources of computations. RF algorithm represents the highest performance with an area under curve (AUC) between 98% and 100% across different keratoconus classes. LR and LDA models provide an AUC varying between 94% and 100% for different keratoconus classes.

However, concerning the comparison of the feature selection algorithms according to the calculated execution time, this work made it possible to classify these algorithms into 3 categories. A first category of the fastest algorithms which are dedicated to execution on personal computers and whose calculated execution time does not exceed 3 minutes, these algorithms are mutual information, ANOVA, embedded, embedded with filter, filter with RFE, RFE, and finally, filter with HRFA algorithms. The second category of these algorithms concerns algorithms for which the calculated execution time varies from 18 minutes to 313 hours, these algorithms require efficient calculators with good hardware configurations, and this category is composed of filter with SFS, SFS, genetic, and filter with SBS algorithms. The third category is composed of algorithms for which the execution time exceeds 300 hours, and the algorithms of this category are SBS algorithm which was applied just on the case of keratoconus classification considering two classes, due to the expensive prediction time it consumed.  Table 6 below resumes different categories of features selection algorithms.

In order to validate the proposed methodology, the adopted process is applied on the database keratoconus [45] composed of 42 features out of 205.  Table 7 below presents a brief description of the used dataset:

In the case of binary classification considering 2 keratoconus classes (normal and keratoconus eyes) and using a subset of six selected variables, the highest performance was achieved, applying 10-fold cross-validation, by RF classifier using genetic selection features algorithm. The best-obtained accuracy was in the range of 93%. In the case of 6 keratoconus classes, the highest performance was provided by the NB model, trained on a subset of 6 selected variables using Boruta [28] algorithm of feature selection. The classification accuracy of this model was 71%.

## 6. Conclusions

In conclusion, the current work represented a comparative study of keratoconus classification performances using different machine learning classifiers. The classification was performed in 2 steps, retaining 2 target classes then considering 4 target classes, applying and without features selection. The obtained results demonstrated that RF algorithm combined to SFS algorithm, which has selected just 10 features, provided a classification accuracy relatively higher than the use of all features, i.e., 446 variables. Given the importance of execution time in addition to classification performance, the use of SFS algorithm has reduced significatively the execution time and has increased classification accuracy by eliminating harmful variables to classification models, hence, the usefulness and the impact of including selection of critical and relevant features to be used in the classification, especially in the case of largest datasets. This work was carried out as part of a project involving machine and deep learning, in the field of ophthalmology, which aims to produce an intelligent system capable of detecting and classifying keratoconus based on the analysis of topographic maps of the eyes.

## Figures and Tables

**Figure 1:** Normal eye (a) and keratoconus eye (b) [6].

**Figure 2:** Feature selection model.

**Figure 3:** Keratoconus classification model.

**Figure 4:** Classification accuracy of different models using all features (a) and applying mutual information (b), ANOVA (c), embedded (d), embedded with a filter (e), and filter with RFE (f) feature selection algorithms.

**Figure 5:** Classification accuracy of different models using RFE (a), filter with HRFA (b), filter with SFS (c), SFS (d), genetic (e), and filter with SBS (f) feature selection algorithms.

**Figure 6:** Classification accuracy of different models using SBS feature selection algorithms.

**Figure 7:** Comparison of classification performance based on the accuracy of different models using all features (a) and applying mutual information (b), ANOVA (c), embedded (d), embedded with a filter (e), and filter with RFE (f) feature selection algorithms.

**Figure 8:** Comparison of classification performance based on the accuracy of different models using RFE (a), filter with HRFA (b), filter with SFS (c), SFS (d), genetic (e), and filter with SBS (f) feature selection algorithms.

**Figure 9:** Comparison of classification performance based on the accuracy of different models using SBS feature selection algorithms.

**Figure 10:** Classification accuracy of different models using all features (a) and applying mutual information (b), ANOVA (c), embedded (d), embedded with a filter (e), and filter with RFE (f) feature selection algorithms.

**Figure 11:** Classification accuracy of different models using RFE (a), filter with HRFA (b), filter with SFS (c), SFS (d), genetic (e), and filter with SBS (f) feature selection algorithms.

**Figure 12:** Comparison of classification performance based on the accuracy of different models using all features (a) and applying mutual information (b), ANOVA (c), embedded (d), embedded with a filter (e), and filter with RFE (f) feature selection algorithms.

**Figure 13:** Comparison of classification performance based on the accuracy of different models using RFE (a), filter with HRFA (b), filter with SFS (c), SFS (d), genetic (e), and filter with SBS (f) feature selection algorithms.

**Figure 14:** Comparison of ROC curves of RF, LDA, and LR algorithms with respect to the normal eyes class (a), forme fruste keratoconus class (b), mild keratoconus class (c), and advanced keratoconus class (d) using the selected variables by applying SFS method.

**Algorithm 1:** Random forest algorithm.

**Algorithm 2:** KNN algorithm.

**Algorithm 3:** LDA steps.

**Algorithm 4:** CART algorithm.

**Table 1:** Summary of previous works in keratoconus classification since 2012.

Authors	Year	Method	Dataset	Inputs	Accuracy	Feature selection
Al-Timemy et al. [8]	2021	SqN, AlN, SfN, MbN	2136 images	N.A	92.2% to 94.8%	N.A
Kamiya et al. [9]	2021	CNN	3390 images	N.A	78.5%	N.A
Jiménez-García et al. [10]	2021	TDNN	743 images	6	N.A	Yes
Kuo et al. [11]	2020	VGG16, InceptionV3, ResNet152	354 images	N.A	93.1%, 93.1%, 95.8%	N.A
Cao et al. [22]	2020	RF, SVM, KNN, LR, LDA, LaR, DT, MPAN	88 eyes	11	87%, 86%, 73%, 81%, 81%, 84%, 80%, 52%	Yes
Lavric et al. [24]	2020	25 classifiers	3151 images	8	62% to 94%	SS, FRank
Velázquez-Blázquez et al. [23]	2020	LR	178 eyes	5	73%	*X* ^2^, Kruskal-Wallis
Lavric and Valentin [12]	2019	CNN	3000	180 × 240 × 3 (images)	99.33%	Yes
Issarti et al. [13]	2019	FNN	851	141 × 141 (images)	96.56%	NCAFS
Salem and Solodovnikov [14]	2019	RF	500	N.A	76%	Yes
Hallett et al. [15]	2019	BNN	124	29	73% (supervised) 80% (unsupervised)	PCA
Luna et al. [16]	2019	BNN	60	16	100%	N.A
Kamiya et al. [17]	2019	CNN	543	6 × 224 × 224 (image)	99.1%	N.A
Yousefi et al. [5]	2018	UnML	3156	420	N.A	PCA NonLinear_tSNE
Hidalgo et al. [18]	2017	SVM	131	25	92.6% to 98%	N.A
Ali et al. [21]	2017	SVM	40	12	90%	N.A
Smadja et al. [19]	2013	DT	372	55	N.A	N.A
Arbelaez et al. [20]	2012	SVM	3502	7	98.2%	N.A

**Table 2:** Studied feature selection methods.

Methods	Algorithms
Filter	Mutual information
	Fast correlation
	ANOVA
	Variance

Embedded	Random forest

Wrapper	Sequential forward selection
	Recursive feature elimination
	Sequential backward selection
	Recursive feature addition
	Genetic

Hybrid	Hybrid recursive feature addition

**Table 3:** Description of different original dataset classes.

Size of original dataset		Class	Number of rows	Percentage size
Number of features	Number of rows			
446	3162	C1	264	8.3%
		C2	2595	82.1%
		C3	221	7%
		C4	82	2.6%

**Table 4:** Classification accuracy of RF model with respect to different feature selection methods.

Model	Feature selector	Keratoconus classification accuracy	
		2 classes	4 classes
Random forest	All features	98.0%	95.32%
	MI	97.15%	90.54%
	ANOVA	97.03%	90.83%
	Embedded	97.63%	91.21%
	Embedded and filter	96.81%	89.79%
	Filter and RFE	97.63%	93.17%
	RFE	97.91%	93.83%
	Filter and HRFA	88.9%	77.9%
	Filter and SFS	97.76%	93.64%
	SFS	98.1%	95.32%
	Genetic	98.04%	94.34%
	Filter and SBS	97.34%	93.71%
	SBS	98.07%	N.A

**Table 5:** Precision, recall, *f*1-score, accuracy, and execution time of different models using different features selection algorithms.

Method	Model	Keratoconus classification using 2 classes					Keratoconus classification using 4 classes				
		Precision	Recall	*F*1-score	Accuracy	Time in second	Precision	Recall	*F*1-score	Accuracy	Time in second
All features	LR	0.97	0.97	0.97	97.38%	1.384256	0.93	0.94	0.93	93.52%	2.281342
	LDA	0.96	0.96	0.96	96.17%	1.949949	0.9	0.9	0.9	89.88%	1.747491
	KNN	0.96	0.96	0.95	95.73%	6.792791	0.91	0.91	0.91	91.37%	5.829261
	CART	0.97	0.96	0.96	96.14%	5.563709	0.92	0.92	0.92	91.49%	6.864419
	NB	0.95	0.93	0.94	93.30%	0.273079	0.89	0.65	0.71	64.80%	0.242261
	SVM	0.93	0.92	0.88	91.88%	9.076491	0.76	0.82	0.75	82.36%	14.471874
	RF	0.98	0.98	0.98	98.00%	16.014512	0.95	0.95	0.95	95.32%	20.485403

Filter and mutual information	LR	0.93	0.93	0.93	93.46%	0.898035	0.81	0.87	0.84	87.35%	2.377594
	LDA	0.97	0.97	0.97	96.93%	0.230103	0.87	0.9	0.87	90.01%	0.092326
	KNN	0.95	0.96	0.95	95.61%	0.259209	0.83	0.87	0.84	87.32%	0.192763
	CART	0.96	0.96	0.96	95.67%	0.180062	0.88	0.88	0.88	87.83%	0.190027
	NB	0.95	0.94	0.94	94.06%	0.060432	0.87	0.8	0.82	79.79%	0.059485
	SVM	0.9	0.92	0.89	91.97%	0.796906	0.77	0.83	0.75	82.58%	1.20752
	RF	0.97	0.97	0.97	97.15%	3.884638	0.89	0.91	0.89	90.54%	4.793544

ANOVA	LR	0.95	0.95	0.95	95.29%	1.03231	0.82	0.88	0.85	88.49%	1.463929
	LDA	0.96	0.96	0.96	96.27%	0.144063	0.86	0.89	0.86	89.28%	0.092706
	KNN	0.95	0.96	0.95	95.57%	0.203406	0.86	0.88	0.87	87.92%	0.186572
	CART	0.96	0.96	0.96	95.61%	0.155927	0.87	0.87	0.87	87.13%	0.165356
	NB	0.95	0.93	0.94	92.85%	0.06592	0.88	0.69	0.74	68.66%	0.067247
	SVM	0.95	0.95	0.95	95.35%	0.628557	0.8	0.86	0.81	85.52%	1.203339
	RF	0.97	0.97	0.97	97.03	3.067386	0.9	0.91	0.9	90.83%	4.246253

Embedded	LR	0.97	0.97	0.97	96.97%	0.772439	0.83	0.89	0.85	88.87%	1.47536
	LDA	0.97	0.97	0.97	97.12%	0.183223	0.88	0.9	0.87	89.66%	0.191917
	KNN	0.96	0.96	0.96	96.33%	0.351021	0.89	0.89	0.88	88.74%	0.198216
	CART	0.97	0.97	0.97	96.55%	0.399475	0.88	0.88	0.88	88.39%	0.343518
	NB	0.96	0.95	0.96	95.16%	0.059198	0.9	0.82	0.85	82.16%	0.061666
	SVM	0.96	0.96	0.96	96.05%	0.745212	0.81	0.86	0.82	86.24%	1.343924
	RF	0.98	0.98	0.98	97.63%	4.735932	0.91	0.91	0.91	91.21%	5.290628

Embedded and filter	LR	0.96	0.96	0.96	96.08%	0.71674	0.8	0.87	0.83	86.62%	1.191328
	LDA	0.96	0.96	0.96	96.11%	0.216366	0.89	0.88	0.85	88.49%	0.059547
	KNN	0.96	0.96	0.96	96.21%	0.185542	0.86	0.88	0.86	88.43%	0.151569
	CART	0.96	0.96	0.96	95.45%	0.084678	0.86	0.86	0.86	85.42%	0.088294
	NB	0.94	0.94	0.94	94.28%	0.06354	0.88	0.89	0.88	88.90%	0.059538
	SVM	0.95	0.95	0.94	94.88%	0.510619	0.8	0.86	0.81	85.80%	0.873448
	RF	0.97	0.97	0.97	96.81%	2.4646	0.89	0.9	0.89	89.79%	2.605076

Filter and RFE	LR	0.98	0.98	0.98	97.63%	0.802103	0.8	0.86	0.82	86.15%	2.173507
	LDA	0.97	0.97	0.97	97.09%	0.180395	0.87	0.9	0.87	89.91%	0.091918
	KNN	0.95	0.96	0.95	95.57%	0.287014	0.83	0.87	0.84	87.29%	0.16819
	CART	0.96	0.96	0.96	96.21%	0.162709	0.9	0.89	0.89	89.28%	0.18652
	NB	0.95	0.94	0.94	94.31%	0.064485	0.87	0.86	0.87	86.31%	0.055916
	SVM	0.9	0.92	0.89	91.97%	0.838237	0.77	0.83	0.75	82.58%	1.209206
	RF	0.98	0.98	0.98	97.63%	3.765689	0.93	0.93	0.93	93.17%	4.597132

RFE	LR	0.94	0.94	0.94	94.37%	0.724412	0.83	0.89	0.85	88.87%	1.428089
	LDA	0.97	0.97	0.97	96.84%	0.173882	0.89	0.9	0.87	89.88%	0.09103
	KNN	0.97	0.97	0.97	97.06%	0.272294	0.9	0.9	0.9	89.98%	0.213538
	CART	0.97	0.97	0.97	96.52%	0.13398	0.91	0.9	0.91	90.26%	0.206897
	NB	0.96	0.96	0.96	95.61%	0.055933	0.91	0.86	0.87	85.52%	0.05992
	SVM	0.96	0.96	0.96	96.14%	0.502924	0.81	0.86	0.82	86.43%	1.160413
	RF	0.98	0.98	0.98	97.91%	3.210188	0.94	0.94	0.94	93.83%	4.381234

Filter and HRFA	LR	0.84	0.92	0.88	91.65%	0.234221	0.7	0.83	0.76	82.89%	1.201195
	LDA	0.84	0.92	0.88	91.65%	0.068874	0.7	0.83	0.76	82.96%	0.063042
	KNN	0.86	0.91	0.88	90.99%	0.173318	0.74	0.81	0.77	80.58%	0.157148
	CART	0.86	0.87	0.86	86.78%	0.078698	0.74	0.76	0.75	76.13%	0.075387
	NB	0.84	0.92	0.88	91.65%	0.060843	0.75	0.83	0.76	83.05%	0.057565
	SVM	0.84	0.92	0.88	91.65%	0.589599	0.7	0.83	0.76	82.99%	1.006607
	RF	0.86	0.89	0.87	88.90%	2.95956	0.74	0.78	0.76	77.90%	3.135792

Filter and SFS	LR	0.96	0.96	0.96	96.30%	0.661703	0.81	0.87	0.84	87.45%	1.456912
	LDA	0.97	0.97	0.97	96.96%	0.092182	0.87	0.89	0.86	89.06%	0.092238
	KNN	0.96	0.96	0.96	95.86%	0.20427	0.84	0.87	0.85	86.75%	0.198333
	CART	0.96	0.96	0.96	95.98%	0.136162	0.9	0.9	0.9	89.98%	0.226029
	NB	0.94	0.94	0.94	94.21%	0.057639	0.89	0.86	0.87	86.12%	0.059771
	SVM	0.9	0.92	0.89	91.97%	0.639869	0.81	0.87	0.83	86.62%	1.280597
	RF	0.98	0.98	0.98	97.76%	3.377056	0.93	0.94	0.93	93.64%	4.575722

SFS	LR	0.98	0.98	0.98	97.60%	0.627829	0.8	0.86	0.82	86.34%	1.447075
	LDA	0.97	0.97	0.97	97.31%	0.150447	0.89	0.9	0.88	89.95%	0.091448
	KNN	0.96	0.96	0.96	96.40%	0.264232	0.9	0.9	0.9	90.01%	0.179493
	CART	0.97	0.97	0.97	97.09%	0.148523	0.91	0.91	0.91	91.33%	0.158256
	NB	0.95	0.94	0.94	94.12%	0.059645	0.91	0.86	0.88	86.09%	0.056018
	SVM	0.96	0.96	0.95	95.89%	0.516274	0.76	0.85	0.8	85.04%	1.071349
	RF	0.98	0.98	0.98	98.10%	3.241881	0.95	0.95	0.95	95.32%	3.702065

Genetic	LR	0.97	0.98	0.97	97.53%	0.660959	0.82	0.88	0.84	87.98%	1.426594
	LDA	0.97	0.97	0.97	96.81%	0.090565	0.9	0.9	0.9	90.36%	0.091082
	KNN	0.97	0.97	0.97	96.81%	0.198013	0.84	0.87	0.85	87.13%	0.183919
	CART	0.97	0.97	0.97	97.12%	0.148974	0.91	0.91	0.91	90.20%	0.191642
	NB	0.96	0.95	0.95	94.75%	0.058466	0.91	0.88	0.89	87.51%	0.055448
	SVM	0.95	0.95	0.95	95.32%	0.636181	0.81	0.87	0.83	86.75%	1.192417
	RF	0.98	0.98	0.98	98.04%	3.51857	0.94	0.94	0.94	94.34%	4.337631

Filter and SBS	LR	0.97	0.97	0.97	96.93%	0.662359	0.81	0.87	0.83	86.88%	1.44051
	LDA	0.96	0.96	0.96	96.24%	0.090107	0.88	0.9	0.87	89.60%	0.091316
	KNN	0.95	0.96	0.95	95.67%	0.192713	0.84	0.87	0.85	86.88%	0.190318
	CART	0.96	0.96	0.96	95.70%	0.14732	0.9	0.9	0.9	90.26%	0.189021
	NB	0.94	0.94	0.94	94.44%	0.055937	0.89	0.83	0.85	82.86%	0.055396
	SVM	0.9	0.92	0.89	91.94%	0.649443	0.81	0.87	0.82	86.53%	1.272575
	RF	0.97	0.97	0.97	97.34%	3.432132	0.94	0.94	0.93	93.71%	4.532753

SBS	LR	0.98	0.98	0.98	97.85%	0.662359					
	LDA	0.97	0.97	0.97	97.31%	0.090107					
	KNN	0.96	0.96	0.96	96.08%	0.192713					
	CART	0.97	0.97	0.97	96.90%	0.14732	N.A				
	NB	0.95	0.94	0.94	93.87%	0.055937					
	SVM	0.95	0.95	0.94	95.07%	0.649443					
	RF	0.98	0.98	0.98	98.07%	3.432132					

**Table 6:** Classification of features selection algorithms based on execution time (hours (h), minutes (min), and seconds (s)) considering 2 and 4 keratoconus classes.

Category	Algorithms	Execution time using 2 classes	Execution time using 4 classes
Category I	Embedded with a filter	1.26 s	1.23 s
	ANOVA	3.59 s	3.59 s
	Mutual information	5.09 s	5.19 s
	Embedded	6.0 s	8.82 s
	Filter with RFE	38.58 s	38.3 s
	Filter with HRFA	1 min 17.58 s	1 min 38.84 s
	RFE	3 min 20.21 s	3 min 19.98 s

Category II	Genetic	9 min 3.07 s	18 min 20.31 s
	Filter with SFS	35 min 54.35 s	45 min 16.61 s
	SFS	3 h 1 min 1.89 s	3 h 31 min 46.47 s
	Filter with SBS	5 h 54 min 3.6 s	7 h 50 min 53.94 s

Category III	SBS	313 h 35 min 16.15 s	N.A

**Table 7:** Description of validation dataset.

Size of original dataset		Class	Number of rows	Percentage size
Number of features	Number of rows			
42	205	C1	82	40%
		C2	40	19.5%
		C3	43	21%
		C4	26	12.7%
		C5	7	3.4%
		C6	7	3.4%

## Data Availability

The current comparative study is based on the public keratoconus dataset of Harvard Dataverse, available in: https://dataverse.harvard.edu/dataset.xhtml?persistentId=doi:10.7910/DVN/G2CRMO.
